RETRACTED

# Machine Vision and Intelligent Algorithm Based on Neural Network

**DOI:** 10.1155/2022/6154453

**Published:** 2022-03-09

**Authors:** Meng Li, Tiebo Sun

**Affiliations:** Department of Mechanical and Electrical Engineering, Jiangsu Food & Pharmaceutical Science College, Huaian 223001, Jiangsu, China

## Abstract

Neural network algorithms and intelligent algorithms are hot topics in the field of deep learning. In this study, the neural network algorithm and intelligence are optimized, and it is used in simulation experiments to improve the target image recognition ability of the algorithm in the machine vision environment. First, this paper introduces the application of neural networks in the field of machine vision. Second, in the experiment, the improved VGG-16 convolutional neural network (CNN) model is applied to metal block defect detection. Experimental results show that the optimized network can classify metal block defects with the maximum accuracy of 99.28%. Then, the intelligent algorithm based on neural network is studied, and the CIFAR-10 data set is taken as the experimental target for training test and verification test. Using BP algorithm, particle swarm optimization algorithm (PSO-BP), and improved neural network algorithm, respectively, the convergence speed of ICS algorithm based on BP neural network is compared. In contrast, ICS-BP algorithm has the fastest convergence speed and converges when the number of iterations is 32, followed by PSO-BP algorithm.

## 1. Introduction

### 1.1. Background

Machine vision technology is widely used in the field of image processing and classification. People began to study new image processing technology and applied neural networks to the field of recognition. Image processing algorithm is an image processing technology and a research hotspot. Artificial neural network (ANN) is an information processing method that simulates human brain neurons. The human brain can process complex information quickly and in parallel, in different environments, and image information can be effectively processed. Robust adaptive image processing can deal with nonlinear noise or impurity data in the image.

### 1.2. Significance

Among various typical deep learning models, CNN performs well. It is more computationally efficient than the fully connected network, and it is easier to adjust the model's hyperparameters and to train on larger-scale data. This article optimizes the VGG-16 model to further improve its processing performance for small sample sets. BP neural network has many advantages that traditional methods do not have, such as autonomous learning ability, self-adaptability, parallel processing, and strong robustness. In the application field of image classification and recognition, BP neural network shows great development potential and prospect. The use of intelligent algorithms based on BP neural network to classify and recognize images provides a new direction and new thinking for the recognition method, which helps image classification be widely used in various fields.

RETRACTED

### 1.3. Related Work

Tanchenko et al. proposed an autonomous calibration algorithm for UAV navigation system. The main comparison is the homography between the visual image system segmented by a computer using CNN and the vector map image. The mathematical and flight experimental results show that the algorithm is effective in navigation applications [1]. Satapathy and colleagues propose a new deep learning model. The learning model is improved with the support of traditional neural convolution neural network. It is proved that using random pool produces better performance than average pool and maximum pool [2]. In Wang and colleague's research, an intelligent hybrid strategy is proposed. This strategy uses *K*-means clustering to establish a feature classification model based on deep convolution neural network [3]. Yin and colleagues mainly propose an intelligent production line network state prediction algorithm for the field of intelligent production, which is based on BP neural network and then improved [4]. Liu and colleagues proposed a new model of concurrent fault identification of wheelset axle box, which was based on an efficient neural network and attention mechanism. Their proposed model improved the extraction ability of various size features [5]. Li and colleagues take an SVM model as the main framework and establish a prediction model combining kernel parameters and parameter optimization. Genetic algorithm, network search, and particle swarm optimization (PSO) are used to optimize the model parameters, which enhances the applicability of the model in practice [6]. Jiang and colleagues proposed an optimized data mining algorithm based on neural network and particle swarm optimization algorithm. First, the kernel function and global discriminant function of distributed data mining are calculated, and the decision model of distributed data mining is established. Experimental results show that the algorithm has high precision and strong convergence [7]. These studies provide some new ideas for this experiment. Tanchenko et al.'s research is very effective for the automatic correction of neural networks, but the selected method is too complicated and the accuracy is not high. Amraei and colleagues' improved method of using random pools is not applicable and has not been used in practical applications. Li and colleagues' optimization experiments with intelligent algorithms have indeed improved the applicability of the model, but at the same time, the performance has not improved.

RETRACTED

### 1.4. Innovation

With the continuous deepening of research, computer machine vision has been continuously developed, and intelligent algorithms have been continuously optimized and innovated. The innovations of this paper are as follows: first, the VGG-16 model is optimized, keeping its convolutional base unchanged, replacing the three connection layers with two new connection layers. The second is to optimize the Cuckoo's intelligent algorithm and introduce the cosine function into the algorithm to make adaptive adjustments to improve the step size and the probability of discovery. The third is to apply the BP neural network to the intelligent optimization algorithm, and its performance has also been verified.

## 2. Methods of Machine Vision and Intelligent Algorithms Based on Neural Networks

### 2.1. Overview of Neural Network Algorithms

#### 2.1.1. Artificial Neural Network

ANNs process distributed and parallel information by simulating animal behavior. It is a network composed of abstract, simplified, and simulated neurons. By adjusting the weights between nodes in the network, a large amount of information in different communication modes can be processed. An important feature of neural network is its self-learning and self-adapting ability, and it is particularly suitable for solving nonlinear problems. “Training” analyzes the mapping between patterns and adjusts the internal weights of the model to make the input-output mappings similar by inputting a set of samples and their corresponding output data. Then use the network to classify the new input, this process is “prediction” [8]. The basic component of the neural network is the neuron, and its structure is shown in Figure 1. The structure contains four parts: input vector, weight, activation function, and output structure. The combination of weights, summation, and activation functions can be collectively called the hidden layer, and the input vector and output become the input layer and the output layer. Multiple layers of neurons can be combined to form a neural network.

Among them, the combination of SUM and *f* is regarded as a hidden neural unit, then the unit is expressed as follows:

(1) $$\begin{array}{c} S⟶f：f\left(\overset{n}{\underset{i=1}{\sum }}a_{i}*w_{i}+b_{1}\right). \end{array}$$

In the formula, *a*_*i*_ is the input vector, *w*_*i*_ is the weight of the input vector, *b*_1_ is the bias term, and *f* is an activation function.

#### 2.1.2. Back Propagation Neural Network

The structure of back propagation neural network is shown in Figure 2. The model framework involves three levels: input level, hidden level, and output level. Units in the same layer have no connection relationship, and units in adjacent layers are connected in one direction [9].

RETRACTED

As the BP neural network processes the nonlinear relationship in a higher-dimensional space and then stores it in a matrix composed of weights, it has good generalization ability and has low requirements for input samples, so it is widely used.

BP neural network uses a supervised learning method, that is, some input and output samples in the network have been obtained in advance. The process is mainly divided into two parts, namely, forward propagation and back propagation. Forward propagation means that after the input layer receives the signal, it calculates the unit value and assigns it to the hidden layer [10]. If it matches, the learning is complete, if it does not match, then backpropagation is performed. According to the original communication path, the reverse calculation is carried out between the actual output and the ideal output, and the neuron weight and displacement of each layer are adjusted by regression method or other algorithms to reduce the signal error [11].

In the BP algorithm, the *S* function is usually used as the output function. In the process of error back propagation, the gradient descent method is used to adjust the weights [12].

Assuming that the output of the *i*th neuron in the previous layer is represented by *O*_i_, the connection weight of neurons *i* and *j* in the current layer is *W*_*ij*_, and the total input of neuron *j* is Sum_*j*_, then

(2) $$\begin{array}{c} {\text{Sum}}_{j}=\sum W_{ij}O_{i},O_{i}=f\left({\text{Sum}}_{j}\right). \end{array}$$

Assume that the number of neurons in the upper layer is represented by *n*, the neural network iteratively operates forward, and *y*_j_ = *O*_*j*_ is the output value of neuron *j* in the output layer, then the average error of the operation is as follows:

(3) $$\begin{array}{c} Er=\frac{\sum_{i=1}^{n}\left(y_{j}-\bar{y_{j}}\right)}{2}. \end{array}$$

Defining the local gradient:

(4) $$\begin{array}{c} \delta_{j}=\frac{\partial Er}{\partial {\text{Sum}}_{j}}. \end{array}$$

Owing to the influence of the weight on the error, it can get,

(5) $$\begin{array}{c} \frac{\partial Er}{\partial W_{ij}}=\frac{\partial Er}{\partial {\text{Sum}}_{j}}\frac{\partial {\text{Sum}}_{j}}{\partial W_{ij}}=\delta_{j}O_{i}. \end{array}$$

Weight correction, generally using the gradient descent method:

(6) $$\begin{array}{c} \Delta W_{ij}=-\eta \delta_{j}O_{i},\\ W_{ij}\left(t+1\right)=W_{ij}\left(t\right)+\Delta W_{ij}\left(t\right), \end{array}$$

Δ*W*_*ij*_ is the change value of the weight, *t* is the number of iterations, *η* is the learning coefficient, and *δ*_*j*_ is the error value between the actual output value and the expected output value.

RETRACTED

BP neural network has a strong nonlinear mapping ability, but the algorithm is easy to fall into a local minimum, and there is a tendency to forget old samples when learning new samples during training. As the number of training increases, the learning efficiency will become lower and the convergence speed will become slower.

#### 2.1.3. CNN

CNNs are mainly used for image processing. Different from the ANN, it has several more layers of structure, which is equivalent to input preprocessing. Its structure is shown in Figure 3, which contains an input layer, a convolutional layer, a pooling layer, a fully connected layer, and an output layer [13]. The fully connected layer is equivalent to the hidden layer.

The convolution operation takes the matrix as the motion matrix of the original image and performs the inner product operation to obtain a matrix smaller than the original image. This process is to intuitively extract some features of the image, such as color, shadows, or contours, as shown in Figure 4.

For a convolution kernel with a size of *m* × *m*, the input image size is *a* × *b*, the step size is *d*, and the filling pixel is *s*, then the output feature map size is a′ × *b*′. Among them, the values of *a*′and *b'* are determined by formulas (7) and (8) [14].

(7) $$\begin{array}{c} a^{\prime }=\frac{a-m+2s}{d}+1, \end{array}$$

(8) $$\begin{array}{c} b^{\prime }=\frac{b-m+2s}{d}+1. \end{array}$$

Multiple convolution kernels perform convolution operations on neurons in the upper layer through weight sharing to obtain a variety of different image features. The more the convolutional layers, the stronger the ability to extract features of the input image. The output of the convolutional layer is as follows:

(9) $$\begin{array}{c} y_{j}^{k}=f\left[\underset{i\in M_{j}}{\sum }\left(y_{j}^{k-1}*\omega_{ij}^{k}+b_{j}^{k}\right)\right], \end{array}$$

where *f*(·) is the activation function, *ω*_*ij*_^*k*^ is the weight of the *i*th eigenvalue of the *k*th layer leading to the *j*th eigenvalue of the *k*th layer, and *y*_*j*_^*k*^ is the eigenvalue of the *j*th output of the *k*th layer, *y*_*j*_^*k*−1^ is the input feature of the *k*th layer, *M*_*j*_ is the set of output feature values of the *k* − 1 layer, and *b*_*j*_^*k*^ is the bias [15].

The pooling layer is periodically interspersed in the middle of the continuous convolutional layer, which is to imitate the human visual system to reduce the dimensionality and abstract image. Pooling uses a feature value to replace a region in the original feature map, which can semantically merge similar features, so the feature vector can be significantly reduced. Pooling functions include methods such as maximum pooling, average pooling, and random pooling [16].

RETRACTED

For the feature map whose input size is *a* × *b* and the pooling area is *m* × *m*, and the step size is *d*, the output feature map size is a′ × *b*′. Among them, the values of *a′* and *b'* are determined by formulas (10) and (11).

(10) $$\begin{array}{c} a^{\prime }=\frac{a-m}{d}+1, \end{array}$$

(11) $$\begin{array}{c} b^{\prime }=\frac{b-m}{d}+1. \end{array}$$

When using the pooling operation, the function learned in a certain layer must be invariant to a small amount of translation of the input, so the pooling layer can greatly improve the statistical efficiency of the CNN model. In many tasks, it is of great significance that the pooling layer can handle inputs of different sizes. For example, when classifying images, the input size of the classification layer must be fixed. By setting the offset size in the pooling area, the classification layer can receive a fixed number of statistical features without having to deal with the initial input size.

The function of fully connected layers is to abstract the features extracted by the convolutional layer, pooling layer, and activation function into high-level semantic features and then map them to the labeled sample space. Each neuron in the fully connected layer is connected to all neurons in the previous layer, which is completed by the dot product operation of the vector. The output of the fully connected layer is as follows:

(12) $$\begin{array}{c} y_{w,b}\left(x\right)=f\left(w^{T}x\right)=f\left(\overset{n}{\underset{i=1}{\sum }}w_{i}x_{i}+b\right), \end{array}$$

*f*(*x*) is the activation function, *w* is the adjustable weight, and *x* is the input of the fully connected layer.

#### 2.1.4. Activation Function

The activation function is to add some nonlinear factors to the neural network, so that the neural network can solve more complicated problems, and the activation function simulates the response of biological neurons. When the accumulation of input signals exceeds the neuron threshold, the neuron is activated and excited, otherwise, it will be inhibited. The commonly used functions in neural networks are Sigmoid function and ReLU function [17].

*(1) ReLU Function*. The ReLU function is a modified linear unit, which can better avoid the gradient saturation effect. The ReLU function is as follows:

(13) $$\begin{array}{c} \text{ReLU}\left(x\right)=\max\left\{0,x\right\}=\left\{\begin{array}{cc} 0, & \;x<0,\\ x, & \;x\geq 0. \end{array}\right.. \end{array}$$

The disadvantage is that it is not centered at 0. During the forward conduction process, if the value of *x* is less than 0, the neuron remains in an inactive state, so that the weight cannot be updated and the network cannot learn.

RETRACTED

As shown in Figure 5, when *x* is greater than 0, the output of the ReLU function has no range limit, and the gradient is 1, which can relatively eliminate the gradient saturation effect of the Sigmoid-type function. At the same time, the ReLU function only needs to pass the derivative of *x* greater than or equal to 0, the weight parameter update speed is fast, and the network sparse expression ability is provided [18]. Improved functions based on the ReLU function include the Leaky_ReLU function and the PReLU function.

*(2) Sigmoid Function*. The expression of the Sigmoid function is as follows:

(14) $$\begin{array}{c} \text{Sigmoid}\left(x\right)=\frac{1}{1+e^{-x}}. \end{array}$$

The function output is shown in Figure 6. The output response range of the Sigmoid function is [0,1], 0 corresponds to the “inhibited state”, and 1 corresponds to the “excited state”. When the input is less than −5 or greater than 5, there is severe gradient saturation. Therefore, it is necessary to prevent parameters from entering this area during network training, which will cause gradient saturation effects and fail to train. The advantage of the sigmoid function is that it is easy to obtain the derivative, but the disadvantage is that it is easy to cause the problem of gradient disappearance due to its soft saturation.

*(3) Tanh Function*. Tanh is a kind of hyperbolic tangent function based on Sigmoid-type function. Similar to Sigmoid, within a certain range, there is also a gradient saturation problem. However, the activation function converges faster, and its output is centered at 0.

(15) $$\begin{array}{c} \text{Tanh}\left(x\right)=\frac{e^{x}-e^{-x}}{e^{x}+e^{-x}}. \end{array}$$

### 2.2. Machine Vision Algorithm Based on Neural Network

#### 2.2.1. CNN-Based Machine Vision Structure

Usually in the field of machine vision, the CNN for processing image tasks is also composed of an input layer, a continuous convolutional pooling structure, a fully connected layer, and a final output layer, as shown in Figure 7.

#### 2.2.2. Machine Vision Image Classification Model Based on CNN

*(1) AlexNet*. AlexNet technology is based on the idea of LeNet and applies the basic principles of CNN to very deep and wide networks. The model has a total of 5 convolutional layers (Conv1 step size is 4, the rest is 1), 3 pooling layers, and 3 fully connected layers. The upper and lower channels are trained in parallel by 2 GPUs at the same time. The main technical content is: the image enters the input layer, goes through the continuous “convolution-pooling” process, then to the fully connected layer, and finally outputs the classification result [19].

RETRACTED

Compared with traditional CNN, AlexNet has several important features: first, it uses data augmentation and dropout strategies to reduce overfitting. The second is to formally apply Relu as the activation function and verify its effect; the third is to propose the LRN layer to normalize the local response; the fourth is to overlap pooling. The sampling step of the pooling layer is smaller than the size of the lower pooling area, which can effectively reduce the information loss caused by the excessively large moving step of the convolution sliding window.

*(2) VGG*. In the structural configuration of the VGG network model, the input image size during training is 244*∗*244, and the only image preprocessing is to subtract the RGB mean value obtained from the training set from each pixel value. Pass through the convolutional layer (3*∗*3), the activation function is ReLU, the convolution step is 1 pixel, and a filter with a smaller receptive field is used. After a series of convolutional layers (usually 13 layers), there are three fully connected layers, and the last layer is the Softmax layer.

The Softmax activation function is as follows:

(16) $$\begin{array}{c} f\left(x\right)=\frac{e^{xj}}{\sum_{k-2}^{k}e^{xk}},\;j=1,\;2,\;3\;\ldots \;,k. \end{array}$$

The calculation formula for convolution with a depth greater than 1 is as follows:

(17) $$\begin{array}{c} y_{i,j}=f\left(\overset{D-1}{\underset{d=0}{\sum }}\overset{S-1}{\underset{n=0}{\sum }}\overset{S-1}{\underset{m=0}{\sum }}W_{d,n,m}X_{d,j+n,j+m}+b\right). \end{array}$$

Among them, *S* is the size of the convolution kernel, *D* is the depth, *b* is the offset, and *W* is the weight of the convolution kernel in the *n* rows and *m* columns of the *d* layer, *x* is the input element, *y* is the feature of the predicted input, and *f*(·) is the ReLU activation function.

Table 1 compares the error rate indicators of various models in the ImageNet classification task. It can be seen from Table 1 that the performance of the VGG algorithm is very good, and the error rate on the Top-1 data set and the Top-5 data set is relatively small, which also provides some reference for subsequent experiments.

### 2.3. Intelligent Algorithm Based on Neural Network

Intelligent algorithms are some novel algorithms or theories in the field of engineering practice. They usually refer to primitive heuristic algorithms for solving optimization problems. Such as genetic algorithm, simulated annealing algorithm, ANN, particle swarm optimization algorithm, there is no unified intelligent algorithm, classification standard, and the most popular multiple solution algorithms belong to this category. The algorithm has multiple solutions in each iteration and has two subcategories: evolutionary algorithm and swarm intelligence algorithm [20]. Evolutionary algorithms are derived from evolutionary theories, such as genetic algorithms and differential algorithms. It guides the selection of the optimal solution through continuous selection, crossover, and mutation. In the global optimization, different probability distributions and existing information are used to generate a new local search range. In the local optimization, the local search is strengthened to achieve the goal of finding the optimal solution.

RETRACTED

#### 2.3.1. Particle Swarm Optimization BP Neural Network Algorithm

The particle swarm optimization algorithm is derived from the study of bird predation problems. Each particle contains all dimensions of the solution to be optimized. After the defined position formula, the position of the particle is continuously updated, and the optimal position of the particle is obtained, so that the global optimal solution can be obtained. Particle swarm algorithm is an easy implementation, fewer parameter settings in the algorithm, and fast convergence speed.

Assuming an *N*-dimensional target search space, a cluster has particles, the position of the *i*th particle is *X*_in_ = (*X*_i1_, *X*_i2_,..., *X*_iN_), the velocity of the *i*th particle is V_in_ = (*V*_i1_, *V*_i2_,..., *V*_iN_). Since in *N*, the particle swarm will update the position to search for individual local extrema, the best position of a single particle is recorded as: *D*Best_in_ = (*D*Bes_i1_, *D*Bes_i2_,..., *D*Bes_iN_). In the process, the particle velocity will also be updated continuously and compare and find the global optimal position *O*Best = (*O*Bes_i1_, *O*Bes_i2_,..., *O*Bes_iN_). The speed and position are updated with:

(18) $$\begin{array}{c} V_{\text{in}}\left(t\right)=V_{\text{in}}\left(t-1\right)+b_{1}r_{1}\left(D{\text{Best}}_{\text{in}}-X_{\text{in}}\left(t-1\right)\right)+b_{2}r_{2}\left(O\text{Best}-X_{\text{in}}\left(t-1\right)\right),\\ X_{\text{in}}\left(t\right)=X_{\text{in}}\left(t-1\right)+V_{\text{in}}\left(t\right). \end{array}$$

Among them, *t* represents the number of iterations, *b*1 and *b*2 are constants, representing learning factors, and *r*_1_ and *r*_2_ are random numbers from 0 to 1.

#### 2.3.2. Improved Cuckoo Algorithm to Optimize BP Neural Network Algorithm

Based on some of the characteristics of cuckoo nurturing offspring and the advantages of Levi's flight, Suash-Deb and colleagues proposed the cuckoo algorithm, which is an algorithm based on the hatching rate of cuckoo eggs, with few parameters and quick optimization. However, the original cuckoo algorithm has many shortcomings, such as insufficient convergence speed and insufficient solution accuracy. Later, researchers proposed more methods to improve the cuckoo algorithm.

*(1) Improvement of Discovery Probability*. The original cuckoo algorithm found that the probability is *P* = 0.25, but according to the actual situation, the discovery probability is dynamically changing, so it is more appropriate to use a variable description. Improving the discovery possibility in the earlier stage of the algorithm helps to increase the diversity of solutions; it is necessary to improve the accuracy and reduce the discovery probability in the late stage of algorithm search, the accuracy should be improved, so the discovery probability should be reduced. The discovery probability is improved as follows:

(19) $$\begin{array}{c} P_{t}=A*P_{\text{initial}},\\ A=\exp\left[\frac{t}{t_{\max}}\right]\cos\left[\frac{t}{t_{\max}}\right]. \end{array}$$

*P*_*t*_ is the discovery probability of the *t*th iteration, the initial discovery probability *P*_initial_ is 0.4, and *A* is the dynamic decrease factor.

*(2) Improvement of Step Size*. Considering in the early stage of the algorithm search, we use a large step size to enhance the search ability of the algorithm; in the later stage of the algorithm search, we use small step length to increase the search precision. The *α*_0_ in the original cuckoo algorithm is a constant which limits the accuracy of the algorithm. Therefore, the cosine function is added to *α*_0_ to make it decrease dynamically. The improved step length formula is as follows:

(20) $$\begin{array}{c} X_{i}^{t}=X_{i}^{t-1}*\alpha_{0}*\left(X_{i}^{t-1}-X_{\text{best}}\right)⊕\text{Levy}\left(\lambda \right),\\ \alpha_{0}=\frac{t_{\text{max}}\cos t-1/t_{\text{max}}}{1000}. \end{array}$$

*X*_*i*_^*t*^ is the position of the *i*th bird's nest in *t* iterations, *t*_max_ is the maximum number of iterations, and cos*t* − 1/*t*_max_ is the function decrement factor.

RETRACTED

## 3. Experiments on Machine Vision and Intelligent Algorithms Based on Neural Networks

### 3.1. Machine Vision Image Target Recognition Experiment Based on CNN

#### 3.1.1. NCC-VGG Optimization

Convolutional network models often have overfitting problems for the training of small sample databases. However, CNNs have an obvious advantage in that they can be reused, which means that image classification models trained on large-scale data sets can also be used in different scenarios, especially in the field of machine vision. This paper proposes an optimization model based on VGG-16 CNN to realize the classification of defect images of metal blocks.

This experiment is pretrained on ImageNet database in advance to solve the overfitting problem. The convolution structure obtained by the VGG-16 model after ImageNet training is shown in Table 2. The image input size is 224*∗*224*∗*3, and the output feature vector is 7*∗*7*∗*512.

The optimized VGG-16 model has two re-established fully connected layers. The training process does not require preprocessing, and the image is directly adjusted to a 224*∗*224 grayscale image. The experiment transforms the VGG-16 model and trains it to classify the defect images of metal blocks. Based on the transfer learning theory, keep the VGG-16 convolutional base unchanged, and replace the previous three fully connected layers (FC) with two new fully connected layers. At this time, only two completely connected layers can be trained to predict the defect category of the metal block. And in terms of activation function selection, as the ReLU function has a potential shortcoming, that is, whether the unit is activated or not, its gradient may be zero during the optimization process, which will lead to a situation where a certain neural unit will never be activated. This paper chooses to use Leaky_ReLU activation function instead of ReLU function to prevent the zero-gradient problem.

#### 3.1.2. Optimized VGG-16 Image Classification Experiment

In the test phase, the image input trained CNN can predict the most likely classification of the output test image. As shown in Figure 8, for the classification of the four types of defects of the metal block (No Defect—Nod, Friction Mark—FM, Blister—BS, and Pit), the prediction results of the convolutional network for the two images are as follows. On the left: the probability of normality is 98.9%, the probability of friction marks is 1.63%, the probability of blistering is 0.47%, and the probability of pit is 0.17%. The probability of judging that the image is defect-free is extremely high. The right one is: the normal probability is 0.21%, the friction mark probability is 96.75%, the blistering probability is 0.49%, and the pit probability is 0.73%. It is very possible to judge that the image belongs to the friction mark defect type. From the image point of view, the classification result is reliable [21]. In actual production, the percentage of classification results can be increased or decreased according to product requirements. If it is set to use the result of the image classification when the probability of a certain category exceeds 90%, otherwise, the image is considered unable to identify the classification output and then turn to the manual detection process.

RETRACTED

The experiment used a total of 7984 images of four defect categories, of which 6344 images were used for the training set, 890 were used for verification, and the remaining 750 were used for testing to test the accuracy of the model's prediction. After 20 iterations of training, the classification results of qualified, and defective products are shown in Figure 9. The results show that the optimized model has excellent performance. The accuracy of training and verification can reach 99.28% and 99.25%, and the accuracy of the test is also as high as 99.25%. And it can be seen from the right of Figure 9 that the training data and verification data loss of the CNN are very low, indicating that the optimized model is fitted.

This article also tried different experimental schemes, using a total of three control CNN models, namely: VGG-16, AlexNet, GoogLeNet, used them to classify the metal block defect images, and gave four classification (classification of no defects, friction marks, blisters, and pits) results. The precision rate and recall rate are also used to evaluate the qualified types, and the results are shown in Table 3. For the four classification results, GoogLeNet showed the best performance. In the test data set, the accuracy rate reached 92.33%, followed by the VGG model. The optimization model proposed in this paper has a great improvement in performance.

For the optimization of other neural network models, the method used is the same as that of VGG-16. After optimization of these two models, the accuracy of the metal block defect detection is relatively high. The classification accuracy rates of Optimized AlexNet and Optimized GoogLeNet are 98.58% and 99.60%, respectively. However, despite the high accuracy, they require more memory and more powerful GPU performance.

### 3.2. Intelligent Algorithm Optimization BP Neural Network Experiment

#### 3.2.1. CS and ICS Comparison Experiment

In this paper, two commonly used test functions, Levy function and spherical function, are used to test the performance of the original cuckoo algorithm and the improved algorithm. The simulation experiment environment is Matlab2014, the number of bird nests is set to 30, the maximum number of iterations is 250, and the two algorithms are run 50 times each. The test function definition is shown in Table 4.

The simulation result is shown in Figure 10. In the comparison of the sphere test function, it can be found that the ICS algorithm curve is always below the CS curve, indicating that the former converges faster and finds the local optimal value faster. And the ICS algorithm reached the optimal value of 0 at the 120th time, and the CS algorithm reached the optimal value at the 185th time. For the Levy test function, the ICS algorithm curve is always below the CS curve, which also shows that the ICS algorithm converges faster. The ICS algorithm reached the optimal value of 0 at the 80th time, and the CS algorithm reached the optimal value at the 145th time. In summary, the improved cuckoo algorithm in this paper converges faster than the original cuckoo algorithm.

RETRACTED

#### 3.2.2. Comparative Experiment of BP, PSO-BP, and ICS-BP

The performance of BP model and two BP neural network algorithms based on intelligent optimization (PSO-BP and ICS-BP) proposed in this paper are compared. Using the CIFAR-10 data set for image classification training and test experiments, which is a data set with data labels. There are 60,000 color images, the size is 32*∗*32, and there are 10 categories. A total of 50,000 images are used for training, and the rest are used for testing, forming a single batch. The verification set is a part of the data set separated from the training set. Setting the number of experiment iterations to 150 times for all types of algorithms. The performance test results of the model are mainly evaluated from the image classification results and convergence speed. The experimental results are shown in Figure 11.

From the BP neural network training convergence graph, it can be concluded that when the number of iterations is about 130, the neural network converges, and the classification effect of the BP neural network is good, but too many iterations will fall into the local optimal problem. From the training convergence graph of the PSO-BP, it can be seen that the PSO-BP algorithm converges at 78 iterations, which improves the performance and efficiency compared to the BP neural network. In the improved cuckoo algorithm optimized BP neural network (ICS-BP) training convergence graph, the number of iterations converges at the 32nd time.

## 4. Discussion

This paper takes artificial intelligence machine vision as the main research object, a theoretical explanation, and a series of experimental research are carried out. The ANN algorithm, BP neural network algorithm, and CNN algorithm are summarized, and the activation functions ReLU, Sigmoid, and Tanh commonly used in neural networks are introduced. In the machine vision mechanism model based on CNN, the commonly used high-performance machine vision image classification models AlexNet and VGG are summarized, and the performance indicators are compared. In the intelligent optimization algorithm, in this paper, the intelligent algorithms of CS and PSO are optimized by BP neural network and propose the PSO-BP and ICS-BP algorithms.

RETRACTED

During the experiment, the VGG model was optimized to make it more suitable for a small image sample set, two new fully connected layers were replaced, and the activation function ReLU was replaced with the Leaky_ReLU function to prevent the zero gradient problem. Then, the optimized VGG-16 model was subjected to image classification experiments, and the results proved that the optimized model has indeed improved the classification performance. For the experiment of intelligent optimization algorithm, firstly compare the Cuckoo algorithm with the improved step size Cuckoo algorithm in the simulation experiment, and then compare the image classification performance of BP algorithm, PSO-BP, and ICS-BP. The results show that among several intelligent algorithms based on BP neural network, ICS-BP has the best performance and the fastest convergence speed.

## 5. Conclusion

Based on related theoretical foundations and human research, an optimized VGG-16 convolution neural network image classification model and a cuckoo optimization algorithm based on BP neural network are proposed. The former is used in the metal block quality testing experiment in industrial production and achieved good results. In addition, the optimized VGG-16 model has better image classification accuracy. ICS-BP has also achieved better results in image classification, and the convergence speed is faster. However, there are many shortcomings in this article. For example, for machine vision, the scope of research is only on image classification, the scope is small, and the functions implemented are relatively single, and there is no design of other areas of machine vision. And with the improvement of the algorithm, the selected neural network algorithm is relatively limited, and no more attempts have been made. It is hoped that future work and research will make further progress in the research of technology and theory.

## Figures and Tables

**Figure 1:** Neuron structure.

**Figure 2:** BP neural network structure.

**Figure 3:** CNN structure.

**Figure 4:** Inner product extraction of image features.

**Figure 5:** ReLU function curve.

**Figure 6:** Sigmoid output function.

**Figure 7:** Image processing CNN structure.

**Figure 8:** Image prediction classification results.

**Figure 9:** Experimental results.

**Figure 10:** Optimal value change graph.

**Figure 11:** Neural network image classification training convergence graph.

**Table 1:** Error rate indicators of each model using the ImageNet data set.

Model	Top-1 validation set	Top-5 validation set	Top-5 test set
VGG	23.7	6.8	6.8
OverFeat	34.0	13.2	13.6
AlexNet	38.1	16.4	16.4
MSRA	27.9	9.1	9.1
GoogLeNet	-	6.7	6.7

RETRACTED

**Table 2:** VGG-16 convolutional structure parameters.

Layer (Type)	Output shape	Parameters
Input	224*∗*224*∗*3	0
Conv1	224*∗*224*∗*64	1728
Conv2	224*∗*224*∗*64	36864
Pool	112*∗*112*∗*64	0
Conv1	112*∗*112*∗*64	73728
Conv2	112*∗*112*∗*64	147456
Pool	56*∗*56*∗*128	0
Conv1	56*∗*56*∗*128	294912
Conv2	56*∗*56*∗*128	589824
Conv3	56*∗*56*∗*128	589824
Pool	28*∗*28*∗*256	0
Conv1	28*∗*28*∗*256	1179648
Conv2	28*∗*28*∗*256	2359296
Conv3	28*∗*28*∗*256	2359296
Pool	14*∗*14*∗*512	0
Conv1	14*∗*14*∗*512	2359296
Conv2	14*∗*14*∗*512	2359296
Conv3	14*∗*14*∗*512	2359296
Pool	7*∗*7*∗*512	0
FC	1*∗*1*∗*4096	102760448
FC	1*∗*1*∗*4096	16777216
FC	1*∗*1*∗*1000	4096000
Total parameters	138M parameters	

**Table 3:** Comparison of test results.

Type	Four categories (%)	Accuracy (%)	Recall (%)
VGG-16	74.76	98.15	95.03
AlexNet	71.24	97.92	68.77
GoogLeNet	92.33	99.16	99.26
Optimized VGG-16	79.73	99.21	99.17
Optimized AlexNet	68.85	98.58	98.06
Optimized GoogLeNet	84.46	99.60	99.49

**Table 4:** Test functions.

	Sphere	Levy
Search area	[−25,25]	[−10,10]
Optimal location	*x∗*= (0,…,0)	*x∗*= (1,…,1)
Optimal value	*f*(*x∗*) = 0	*f*(*x∗*) = 0

## Data Availability

Data sharing not applicable to this article as no data sets were generated or analysed during this study
